# Multi-Agent-Based Film Editing Collaboration System

**DOI:** 10.1155/2022/1327620

**Published:** 2022-07-01

**Authors:** Along Liang

**Affiliations:** Xi'an Shiyou University, Shaanxi 710065, Xi'an, China

## Abstract

In order to realize the effective cooperation between editor agents in the film and television editing collaboration system, it is analyzed that the state change of the film and television editing and production process is affected by the cross influence of multiple factors. A single agent can no longer satisfy the current film and television production. From the point of view of system theory, this article constructs the learner agent in the film and television editing system by introducing a new cooperation mechanism—the multi-agent collaborative system model. Collaboration and cooperation between multiple agents and the reinforcement learning between multiple editor agents are realized based on the film and television editing system between multiple agents. The operation mechanism of the separate organization is organized together, cooperates with each other and works in harmony to complete the collaborative effect of the film and television editing system, and can improve the interaction efficiency between the editor agents. Agent film and television editing's cooperative learning approach allows for successful collaboration among editor agents. The Bayesian technique is utilized in this study to assess the likelihood of effective cooperation between two agents, and a trust model based on this method is presented, making up for the shortcomings of the existing collaborative learning system. The multi-agent collaboration system will be utilized for production in the film and television editing collaboration system. Many of the movie's scenes and segments are created using computer technology special effects, giving viewers a very unique experience and a feast for the eyes and ears.

## 1. Introduction

The most basic and fundamental technology in film and television editing is fine-tuning the video material and pictures that have been shot in the video and connecting the meaningless fragments into a summary with a plot that follows a certain logic. Multi-agent collaboration is a hot topic in distributed artificial intelligence research in the realm of film and television editing, as well as a hot topic in multi-agent collaboration system technology. In the realm of film and television editing, research on multi-agent collaboration systems now focuses mostly on interaction in a multi-agent system. Each agent can be regarded as an autonomous entity (such as a software program or robot). The agency can use multiagent system and video special effects, including special effects sound and color correction, to produce unique visual effects, such as smoke, water, fire, fog, explosion, and collapse, and other effects that cannot be captured by video, so as to complete complete film and television works. After adding subtitles, actors, producers, and other information, the editor combines the produced files with the produced video special effects to form a movie with coordinated sound, picture, and rhythm and finally render and output it as a movie.

Video editing includes professional skills in video shooting, video special effects, etc. The scope of film and television editing includes film and television advertisements, feature films, product introductions, conferences, lectures, training, sports meetings, large- and medium-sized schools, etc., video shooting and production includes post production, planning activities, film and television program planning, film, and television work, video shooting and production includes advertising planning, agency, publishing, advertising film shooting, advertising design and production, graphic design and production, organizing large‐ and medium-sized cultural exchange activities, etc. The interaction between agents can be collaborative or selfish. Collaboration is the key concept to distinguish multi-agent systems from distributed computing, object-oriented systems, and expert systems. How to carry out in a multi-agent system? Effective prevention and cooperation of withering is a difficult problem to achieve. Theoretical analysis shows that if a learning mechanism is introduced in a cooperative multi-agent system, each agent can effectively accomplish the common goal by coordinating its own behavior through learning. Therefore, learning in the cooperative process has received more and more researchers' attention. Game theory researchers have extensively studied the role of learning in the process of cooperation, such as virtual game “and Bayesian optimal response method,” which can achieve better coordination in a simple gaming environment. However, these models assume that the agent can completely observe the actions taken by other agents during the interaction process. In practical applications, due to the dynamic nature of the environment and the randomness of actions, this assumption is usually not established. At this time, the editing and collaboration systems in cinema and television are also constantly evolving. In film and television editing, a variety of technologies are employed. A great number of magnificent works, which are high-quality completed items made by employing synthesis technology, have also been produced in such a multi-agent system.

Nowadays, society is developing, technology is making continuous progress, and the film and television industry has been greatly impacted by technology. With the continuous advancement and development of science and technology, the editing of film and television works has gradually undergone new changes, and the traditional and outdated editing concepts such as “pre-shooting” have long been abandoned. Based on the multi-agent film and television editing collaboration system, we can regard multi-agent film and television editing as secondary creation and even interpret it as secondary shooting. The effective combination of film and television editing and film and television shooting can get rid of the shackles of the previous and subsequent stages. Based on the editing perspective of the multi-agent collaborative system, we can regard film and television editing as a relatively complete multi-agent autonomous generation process and run through the editing in all aspects of film and television work creation. In the process of horizontal editing, it is necessary to coordinate the rhythm of sound and picture and the role of shot combination in film and television production. It is necessary to pay attention to the interaction between the director and the camera lens, pay attention to the harmony between the structure and the picture, and finally form a film and television clip by integrating these materials, so as to produce a high-quality film and television work. First, various materials can be freely zoomed, rotated, and moved in various types of digital editing software, and one or even thousands of virtual cameras can be set up to perform panning, pushing, pulling, etc. Shift and other operations will eventually obtain special shooting visual effects that were not obtained during the original shooting, which will bring a strong visual impact. At this time, post-editing is required. Second, the multi-layer control functions and selection functions in the multi-agent film and television editing collaboration system software can make the synthesized images show various virtual reality, light and shade changes, etc., so as to successfully realize the multi-layer depth of field control that cannot be achieved in the shooting stage. Local exposure has multilevel and other control effects, so that the audience can enjoy and experience a more vivid visual feast. Editing is a second shot in the three-dimensional creative realm. Based on today's digital technology, we can only make full use of diverse materials with this idea, and then we can expand our wings of creativity, edit, and produce higher quality and greater effect film and television goods with this concept.

The present film and television production can no longer be met by a single agency. Therefore, this article introduces a novel cooperation mechanism, the multi-agent collaborative system model, to design the learner agent in the film and television editing system. The film and television editing system among numerous agents facilitates collaboration and cooperation among agents, as well as reinforcement learning among editors. The distinct organization's operation mechanisms are grouped together, collaborate with one another, and function in harmony to complete the collaborative impact of the film and television editing system, as well as increase the interaction efficiency among editor agents.

The remaining sections and subsections of the paper are arranged as given below.

Bayesian method-enabled reliability evaluation model is reported in upcoming section where basic components are described first followed by a detailed and thorough explanation of the scheme especially from the current domain perspective. Formation of the multi-agent collaborative system is reported in Section 3 of the paper which is followed by a summarized form of the complete work presented in this paper.

## 2. Reliability Evaluation Model Based on Bayesian Method

Reliability is defined as the process of establishing whether or not an existing system or entity has met a predetermined degree of operational dependability.

### 2.1. Basic Concepts

In the interpersonal network, trust relationship is the core of interpersonal relationship, trust is the evaluation of the credible behavior of a specific individual, and the credibility of an individual often depends on the recommendation of other individuals [1–3]. The multi-agent system is very similar to the interpersonal network, which is shown in the following:

- When an agent in a network cooperates with other agents, it will leave information indicating its behavior characteristics.
- The agent has a sufficient choice of cooperation objectives.
- The actor has an obligation to give recommendation information for other agents in the network [4].

As a result, agents may perform trust evaluations based on the actions of cooperating parties, and they can also share and distribute assessment information to determine the target agent's trustworthiness, guiding agents' cooperative decision making. In this work, “trust” in a multi-agent system is defined as the assessment of a target agent's ability to offer services (resources) based on the consistency of the agent's behavior in a given context, including the observation of the agent's previous conduct and other agents' opinions on it [5]. Trust is within a certain range and changes dynamically according to multiple collaborations between agents. Generally speaking, the trust relationship is not absolute, but dynamic. A trusts B's ability to provide a certain service. With the increase in the number of collaborations with B, A will gradually change and adjust the credibility of B according to the success of the collaboration, forming A's direct trust in B. In addition, trust also has a recommendation relationship [6]. When the agent has not communicated with an agent directly before, it can only rely on the recommendation information provided by other agents as a reference and judge the recommendation information according to its own strategy. The above analysis of the attributes of the trust relationship provides the necessary basis for the trust evaluation and the design of the trust computing model [7].

In a multi-agent system, there may be direct cooperation between one agent and other agents, and there may also be intermediate agents that cooperate with both parties. Accordingly, Bayesian analysis is based on subjective probability, which is an opinion and a measure of reasonable belief. It is a measure of someone's belief (or view) of the probability that a particular event will occur, that is, how likely he believes or thinks the event will occur. The degree of this belief is a kind of belief, which is subjective, but it is set based on experience, knowledge of various aspects, and understanding of the objective situation, using relevant information to analyze and reason and make comprehensive judgments. Therefore, the Bayesian method is very suitable for the assessment of trust.

In the same sense, trust is difficult in multiagent systems. In the system, there are two agents. This study uses word of mouth to express the possibility of effective cooperation. If *z* and Y collaborate directly, we may try to predict the likelihood of direct cooperation succeeding, which is known as direct credibility assessment and is given in percent [8]. At the same time, if there is one or more intermediate agents w (also known as recommended agents) between *Z* and *Y*, *W* can be used as the recommended agent to establish a link, and the relationship between *Z* and *Y* can be obtained directly through *W*. The recommendation credibility evaluation is the collection of information regarding a successful partnership. Combine these two probabilities to obtain the overall credibility evaluation of successful collaboration, which is given by the following formula:

(1) $$\begin{array}{c} \overset{\wedge }{\theta }=w_{1}\overset{\wedge }{\theta_{dt}}+w_{2}\overset{\wedge }{\theta_{rt}}, \end{array}$$

where W1 and W2 are the weights that determine the importance of the two kinds of credibility, satisfying the conditions *w*_1_, *w*_2_ ∈ [0,1] and *w*_1_+*w*_2_=1. Its value is determined by the subjective factors of the agent. For example, an agent who believes that his direct experience is better than the recommendation of others will choose *w*_1_ > *w*_2_.

### 2.2. Direct Credibility Assessment

For the direct credibility of the collaboration between two agents, the Bayesian analysis is used in this paper to obtain the estimated value. Suppose there are two agents *x* and Y in a multi-agent system; if a binomial event (success/failure) is used to describe the collaboration result between them, when *n* collaborations between *x* and Y occur, the number of successes is *u*, and the number of failures is *v*, and the direct credibility $\overset{\wedge }{\theta_{dt}}$ is defined as the probability that the *n*+1th collaboration succeeds. Then, the posterior probability of successful cooperation between *x* and Y obeys the Beta distribution, and its density function is

(2) $$\begin{array}{c} \text{Beta}\left(\theta |u,v\right)=\frac{\Gamma \left(u+v+2\right)}{\Gamma \left(u+1\right)\Gamma \left(v+1\right)}\theta^{u}{\left(1-\theta \right)}^{v}. \end{array}$$

(3) $$\begin{array}{c} \overset{\wedge }{\theta_{dt}}=E\left(\text{Beta}\left(\theta |u+1,v+1\right)\right)=\frac{u+1}{u+v+2}, \end{array}$$

where 0 < *θ* < 1 and parameters *u*, *v* > 1.

The value of direct credibility is connected to the success probability of the target agent delivering services in the past and the total number of partnerships, according to formula (3), and it also indicates the target agent's capacity to provide consistent service quality in the network. Although formula (3) specifies the direct reliability calculation method [9], this technique has two flaws: first, an agent may not have worked with the target agent, making it impossible to assess the agent's dependability; second, an agent may only have a few experiences working with the target agent, which is inadequate. It is used to assess the target agent's believability. In both cases, due to lack of sufficient evidence (observation), use $\overset{\wedge }{\theta_{dt}}$ directly. It is no longer suitable to estimate the true reliability of the target. Therefore, the collaboration records of other agents to the target agent must be collected [10], and the credibility calculated in this way is the recommendation credibility mentioned earlier in this paper.

### 2.3. Recommendation Reliability Assessment

Since the mechanism of recommendation trust is formed by the direct cooperation of two or more categories, the above method can still be used for its evaluation.

Let the cooperation between agents *x* and Y and between *z* and Y in the multi-agent system be independent; then, the number of cooperation is *n*_1_ and *n*_2_, the number of success is *u*_1_ and *u*_2_, and the number of failure is *v*_1_ and *v*_2_. Then, the estimation of the recommendation trust value of *x* through *z* is

(4) $$\begin{array}{c} \overset{\wedge }{\theta_{rt}}=E\left(\text{Beta}\left(\theta |\left(u_{1},v_{2}\right),\left(u_{2},v_{2}\right)\right)=\frac{u_{1}+u_{2}+1}{n_{1}+n_{2}+2}\right). \end{array}$$

When there is more than one recommended agent, it is not difficult to generalize as shown in the following formula:

(5) $$\begin{array}{c} \overset{\wedge }{\theta_{rt}}=\frac{\sum u+1}{\sum \left(u+v\right)+2}. \end{array}$$

### 2.4. Analysis of the Trust Relationship between Agents

The relationship can be divided into four types based on whether there is direct cooperation between any two agents and whether there are two aspects of recommending agents [11]. If dt = 1 (or 0), it means that there is (or is not) direct cooperation between agents *x* and Y, and rt = 0 (or 1) means that there is (or is not) recommending agent between *x* and Y; then, these four variables must be true. TR is a basic two-tuple representation of the trust relationship (dt, rt). This research examines the assessment of overall believability in each of these four scenarios one by one.

(1) TR (dt, rt) = (O, 0). In this case, there is no direct cooperation between *x* and Y, and there is no recommended agent. Therefore, the prior distribution of *θ* should choose the uninformative prior distribution U(0,1), that is, Beta(1,1). Thus, the overall credibility (i.e., the estimated probability of successful collaboration) $\overset{\wedge }{\theta }=1/2$.
(2) TR(dt, rt)=(1, 0). That is, there is only direct cooperation between *x* and Y, and the estimated value of the probability of successful cooperation can be obtained by formula (3).
(3) TR(dt, rt)=(0, 1). In this case, there is a recommendation agent between *x* and Y, but there is no direct cooperation. Therefore, the direct reliability *θ*_*dt*_ still adopts 1/2, and the recommended reliability *θ*_*rt*_ is calculated by formula (5). Finally, the combination is carried out by formula (1), that is,
  (6) $$\begin{array}{c} \overset{\wedge }{\theta }=w_{1}\times \frac{1}{2}+w_{2}\times \frac{\sum u+1}{\sum \left(u+v\right)+2}. \end{array}$$
(4) TR (dt, rt) = (1, 1). That is, there is direct cooperation between *x* and Y, and there is a recommendation agent. When calculating the reliability, use formula (1) to calculate, where *θ*_*dt*_ and *θ*_*rt*_ are given by formulas (3) and (5), respectively, namely,
  (7) $$\begin{array}{c} \overset{\wedge }{\theta }=w_{1}\times \frac{u+1}{u+v+\_2}+w_{2}\times \frac{\sum u+1}{\sum \left(u+v\right)+2}. \end{array}$$

Note that $\overset{\wedge }{\theta }$ is the trust value of agent *x* to Y, *N*_*x*_ is the set of neighbor agents of *x*, and *M*_*x*_ is the set of agents for which *x* has its trust record. If the value is the smallest and *y* ∈ *M*_*x*_ − *N*_*x*_, *N*_*x*_, the link with *z* is replaced with the link of Y; if the trust value of *z* in *y* ∈ *N*_*x*_, *M*_*x*_ − *N*_*x*_ is the largest and $\overset{\wedge }{\theta }>\overset{\wedge }{\theta_{z}}$, the link with *z* is replaced with the link of Y.

## 3. Formation of Multi-Agent Collaborative System

### 3.1. Establishing a Multi-Agent Collaboration System

In this paper, the probability of successful cooperation between agents is taken as the index of trust, and a multi-agent cooperation system based on trust mechanism is obtained accordingly. Any agent in the system may become the object of the agent's next cooperation, and each entity in the system is trusted to different degrees and is likely to become the cooperation object in the future cooperation [12, 13]. Therefore, a relatively stable multi-agent cooperative system can be formed after a certain period of time.

Based on the above ideas and with the help of the node link mechanism in the P2P overlay network, this paper presents a link update algorithm based on the trust mechanism to form a multi-agent cooperative system [14], so that the agents in the system can be established more easily with the agents with stronger service capabilities. Close collaboration is shown in Figure 1.

The distributed collaborative film and television editing system consists of a core film and television editor and multiple collaborative film and television editors scattered on several systems; each film and television editor has several film and television editors within it. It is a competitive partnership between the film and television editors (hope to cooperate, but always strive to maximize their own benefits) [15]. Simultaneously, there is mutual reliance (collaborative film and television editing provides the necessary film and television editing for the core film and television editor). Within the film and television editors' community, there is a cooperative connection (the goal is to maximize the overall interests of the agent). Observing the collaborative system, analyzing the business, collaborating with other collaborative film and television editors to get assignments, and dealing with the dynamic incoming task needs are all significant duties of the collaborative film and television editor. Distribute among the agent's film and television editors.

The main responsibility of the film and television editor is to perform the tasks assigned by the cooperative film and television editor. Communicate and work with other film and television editors when necessary. The collaborative system is triggered by tasks to generate film and television editing requirements [16], and each collaborative film and television editor must deal with dynamic logistics tasks at any time. Film and television editors play a central role in the collaborative system, and their main responsibility is to find opportunities for collaborative systems and transform them into tasks that meet the requirements of the opportunities. For small tasks, film and television editors can complete them by themselves, while for tasks that require multiple resource support or time constraints and large logistics, multiple editors are required to cooperate to solve them. At this time, film and television editors will search for editors who meet the requirements through the Internet and implement all tasks one by one until each task is committed. The editor plays the role of a subcontractor in the collaboration system. On the one hand, it sends out task requests to the film and television editor through the network, and on the other hand, it analyzes the tasks issued by the film and television editor, and according to its own ability, it can perform tasks in numerous tasks [17, 18]. In order to solve the problem of film and television editing in the above-mentioned collaborative system, many agents are introduced. Independent and autonomous agents are used to represent film and television, respectively. Edit and agent form a new collaboration system. When the agent receives a new task, it generates one or several task agents. The task agent and the SAgent determine the relationship between each subtask and each film and television editor through cooperation. The management agent is the core agent of the system, which is equivalent to the role of the system administrator, and manages the various agents that make up the collaborative system; at the same time, it is also responsible for information interaction with editors and task release. Management agent also manages the communication between different agents.

### 3.2. Establishment of Multiagent Cooperative System

Film and television editors not only depend on how to choose partners but also need to weigh and analyze whether to join the new cooperation system. For cooperative systems, potential member agents need to adjust their strategies continuously during the negotiation process and choose a coalition structure that is most beneficial to them. Feng Wen described the negotiation process of the cooperative system by using a multi-agent multi-stage negotiation model, which can ensure the maximization of the global benefit of the cooperative system. The selected members are the most competitive, and the member agents can obtain satisfactory benefits, which truly reflects the “win-win” feature. Collaborative process is based on multiagent. Assuming that the film and television editing request agent receives the task *T* that needs to be completed by A type of agent, the task agent on the one hand queries the agent that can complete each subtask from the facilitator's ability and ANS; on the other hand, the task agent publishes tasks to the Internet. If for each type of subtask, there is at least one agent corresponding to it in the returned agent list and Internet, then start the multi-stage negotiation process [19]. The first stage is the negotiation between the film and television editor and the potential editor, and the film and television editor asks the potential editor to give an initial specification suggestion for the task. The film and television editing system evaluates the proposal. The second stage is a multi-lateral negotiation between potential editors. It can be known from the multi-lateral negotiation process that the top ranked in the set list has priority as a potential alliance [20, 21]. This is consistent with the agent's goal of pursuing the maximum benefit of the individual. Therefore, the negotiation process can not only ensure the maximization of the global benefits of the collaboration system but also enable the agents to participate in the collaborative production benefits, which truly reflects the goal of perfecting the film and television editing collaboration system.

## 4. Conclusion

Multi-agent systems have a significant effect on various application domains including editing cooperation system for the film and television. The film and television editing cooperation system investigated in this study employs a multi-agent mechanism to solve the editing and synthesis skills and various agents to realize the system's tasks. Each agent addresses local difficulties in accordance with the purpose of film and television editing technology, and they can work together to meet the overall deadline. The multi-agent film and television editing collaboration system provides a significant reference value for the administration of diverse agents in the film and television business, thanks to the research solution of the multi-agent film and television editing collaboration system.

In future, the proposed model could possibly be extended to various other domains and could be combined with other approaches.

## Figures and Tables

**Figure 1:** Link update based on multi-agent collaboration system.

## Data Availability

The data used to support the findings of this study are available from the corresponding author upon request.
